# Deep Learning-Based Image Feature with Arthroscopy-Aided Early Diagnosis and Treatment of Meniscus Injury of Knee Joint

**DOI:** 10.1155/2021/2254594

**Published:** 2021-09-17

**Authors:** Zijian Li, Shiyou Ren, Xintao Zhang, Lu Bai, Changqing Jiang, Jiangyi Wu, Wentao Zhang

**Affiliations:** Department of Sports Medicine and Rehabilitation, Peking University Shenzhen Hospital, Shenzhen 518036, China

## Abstract

The aim of this study is to explore the clinical effect of deep learning-based MRI-assisted arthroscopy in the early treatment of knee meniscus sports injury. Based on convolutional neural network algorithm, Adam algorithm was introduced to optimize it, and the magnetic resonance imaging (MRI) image super-resolution reconstruction model (SRCNN) was established. Peak signal-to-noise ratio (PSNR) and structural similarity (SSIM) were compared between SRCNN and other algorithms. Sixty patients with meniscus injury of knee joint were studied. Arthroscopic surgery was performed according to the patients' actual type of injury, and knee scores were evaluated for all patients. Then, postoperative scores and MRI results were analyzed. The results showed that the PSNR and SSIM values of the SRCNN algorithm were (42.19 ± 4.37) dB and 0.9951, respectively, which were significantly higher than those of other algorithms (*P* < 0.05). Among patients with meniscus injury, 17 cases (28.33%) were treated with meniscus suture, 39 cases (65.00%) underwent secondary resection, 3 cases (5.00%) underwent partial resection, and 1 case (1.67%) underwent full resection. After meniscus suture, secondary resection, partial resection, and total resection, the knee function scores of patients after treatment were (83.17 ± 8.63), (80.06 ± 7.96), (84.34 ± 7.74), and (85.52 ± 5.97), respectively. There was no great difference in knee function scores after different methods of treatment (*P* > 0.05), and there were considerable differences compared with those before treatment (*P* < 0.01). Compared with the results of arthroscopy, there was no significant difference in the grading of meniscus injury by MRI (*P* > 0.05). To sum up, the SRCNN algorithm based on the deep convolutional network algorithm improved the MRI image quality and the diagnosis of knee meniscus injuries. Arthroscopic knee surgery had good results and had great clinical application and promotion value.

## 1. Introduction

The knee joint is the largest, most complex, and weight-bearing main joint in the human body. Patients with tibial plateau fractures are often accompanied by meniscal injuries, and the incidence is about 50% [1]. Meniscus injuries are difficult to repair themselves, which is a difficult and urgent problem in orthopedic treatment. Meniscus injuries are often diagnosed by arthroscopy, knee ultrasound, CT, and magnetic resonance imaging (MRI). Arthroscopy is the gold standard for meniscus diagnosis, but it is invasive and increases the probability of infection in patients [2]. The diagnostic accuracy of B-ultrasound for knee joint meniscus injury is not high [3]. CT cannot correctly grade the diagnosis. MRI has the characteristics of noninvasiveness, nonradiation, high soft tissue resolution, and high specificity. Moreover, MRI has high sensitivity and specificity to the injured area, so MRI has become an important method for knee joint injury following arthroscopy [4]. However, affected by the resolution of MRI images, the false positives and false negatives of meniscus injury diagnosis are relatively high.

MRI images are susceptible to noise pollution, resulting in distortion of MR images [5]. At present, MRI images are often processed by filtering-based denoising methods, but the image information is lost seriously in the denoising process, and additional noise may be introduced [6]. Convolutional neural networks have achieved very good results in natural image processing. At present, some scholars have applied them in the field of medical images. High-resolution MRI images can be obtained after being processed by super-resolution reconstruction algorithm [7]. Kobayashi et al. [8] pointed out that the image resolution processed by the three-layer convolutional neural network (CNN) (super-resolution CNN, SRCNN) was significantly improved. However, there are still obvious misdiagnosis and missed diagnosis in the diagnosis of clinical diseases, which need to be further improved.

In summary, the resolution of MRI images requires to be further improved. SRCNN based on deep CNN algorithm should be further optimized to increase its image quality. Therefore, SRCNN was optimized based on the deep CNN algorithm in this research. Patients with knee meniscus injury were taken as the research object to explore the diagnostic value of MRI images of deep CNN algorithm for meniscus injury. Moreover, the clinical effect of arthroscopic surgery based on MRI images in knee meniscus injuries was evaluated to provide guidance for the treatment of knee meniscus injuries.

## 2. Materials and Methods

### 2.1. Research Objects and Grouping

Sixty patients with knee meniscus injury who were admitted to the Orthopedics Department of our hospital from August 2019 to December 2020 were selected as the research objects. The age range was 18–70 years old, and the average age was (48.54 ± 5.46) years old. Among them, 41 were males and 19 were females. The meniscus injury time was seven days to five years, and the average injury time was (2.24 ± 1.04) years. There were 37 cases on the left and 23 cases on the right knee. All patients had no history of knee surgery and received knee MRI and knee arthroscopy during examination and treatment. Inclusion criteria were as follows: (i) age> 18 years; (ii) MRI examination showing meniscus injury, which was confirmed by knee arthroscopy; (iii) those who were hospitalized in time and can receive surgery; and (vi) those with no contraindications to surgery. Exclusion criteria were as follows: (i) patients with other fractures or severe system diseases; (ii) patients with meniscus congenital diseases or developmental abnormalities; (iii) patients combined with knee joint infection, tuberculosis, and so on; and (iv) meniscus injury caused by severe bone and joint disease. The experimental procedure had been approved by the hospital ethics committee, and all subjects included in the study had signed the informed consent form.

### 2.2. MRI Image Super-Resolution Algorithm Based on Deep CNN Algorithm

The convolutional layer of the deep CNN (DCNN) is mainly responsible for extracting features from the input data [9], and the extracted feature map *X*_*l*_ output by the first layer is expressed as follows:

(1) $$\begin{array}{c} X_{l}=X_{l-1}⊙A_{l}+b_{l}, \end{array}$$

where *X*_*l*−1_ is the output of the *l*-th layer, ⊙ is the convolution operation, *A*_*l*_ is the convolution layer parameter, and *b*_*l*_ is the bias. The activation function in DCNN can improve the expressive power of the entire network by introducing nonlinear operations [10]. The ReLU function can avoid the disappearance of the gradient when the input is saturated [11]. The ReLU function is expressed as follows:

(2) $$\begin{array}{c} g\left(x\right)=\left\{\begin{array}{cc} x, & \left(x\geq 0\right),\\ 0, & \left(x<0\right). \end{array}\right. \end{array}$$

The training goal of DCNN is minimizing the loss function of the network [12]. The commonly used loss functions include mean square error loss function, cross-entropy loss function, and log-likelihood loss function. The mean square error loss function is expressed as follows:

(3) $$\begin{array}{c} B=\frac{\sum_{i=1}^{m}{\left(y_{i}-\hat{y_{i}}\right)}^{2}}{m}. \end{array}$$

The cross-entropy loss function is expressed as follows:

(4) $$\begin{array}{c} B=\frac{1}{m}\sum_{i=1}^{m}y_{i}\log\left[h_{0}\left(x_{i}\right)\right]+\left(1-y_{i}\right)\log\left[1-h_{0}\left(x_{i}\right)\right]. \end{array}$$

The log-likelihood loss function is expressed as follows:

(5) $$\begin{array}{c} B=-\sum_{i=1}^{m}y_{i}\ln\;h_{0}\left(x_{i}\right), \end{array}$$

where *m* is the number of input samples, $\hat{y_{i}}$ is the corresponding model output of *x*_*i*_, *y*_*i*_ is the corresponding target output, and *h*_0_(*x*_*i*_) is the corresponding model probability output of *x*_*i*_.

The DCNN-based super-resolution reconstruction algorithm (SRCNN) mainly includes image feature extraction, nonlinear mapping, and image reconstruction when processing low-resolution images. After the low-resolution images go through image data preprocessing, DCNN feature extraction, and nonlinear mapping and image reconstruction modules in the SRCNN module, a high-resolution MRI image is obtained. SRCNN processing flow for low-resolution images is shown in Figure 1.

Before low-resolution MRI image processing, it is necessary to perform preprocessing such as normalization, low-resolution image generation, image feature extraction, and data enhancement. The data types of MRI images are mostly 32-bit floating-point numbers. The calculation method for normalizing MRI images is as follows:

(6) $$\begin{array}{c} C_{i}^{\prime }=\frac{C_{i}}{\max\left(C_{i}\right)}, \end{array}$$

where *C*_*i*_ is the matrix of the original *i*-th MRI image and *C*′ is the normalized MRI image of the *i*-th image.

The neural network training process is divided into forward propagation process and backpropagation process. The forward propagation process uses the network input and existing parameters to calculate the network output. The backpropagation process first calculates the loss based on the network output and then transmits the loss back to each node in the network, thereby updating the weight value of each node [13]. For the simplest gradient descent algorithm, the weight update process is expressed as follows:

(7) $$\begin{array}{c} \left\{\begin{array}{c} \omega_{i+1}=\omega_{i}-\alpha \text{d}\omega ,\\ e_{i+1}=e_{i}-\alpha \text{d}e, \end{array}\right. \end{array}$$

where *ω*_*i*_ is the current weight, d*ω* is the gradient of the loss function to *ω*, *ω*_*i*+1_ is the updated weight, *e*_*i*_ is the current bias term weight, d*e* is the gradient of the loss function to *e*, *e*_*i*+1_ is the updated bias term weight, and *α* is learning rate.

The momentum gradient descent algorithm is a common algorithm for parameter update in the network, and its update parameters are expressed as follows:

(8) $$\begin{array}{c} \left\{\begin{array}{c} D_{\text{d}\omega }=\beta D_{\text{d}\omega }+\left(1-\beta \right)\text{d}\omega ,\\ D_{\text{d}e}=\beta D_{\text{d}e}+\left(1-\beta \right)\text{d}e,\\ \omega_{i+1}=\omega_{i}-\alpha D_{\text{d}\omega },\\ e_{i+1}=e_{i}-\alpha D_{\text{d}e}, \end{array}\right. \end{array}$$

where d*ω* and d*e* represent the current gradients, *D*_d*ω*_ and *D*_d*e*_ represent momentums, and *β* is a self-set hyperparameter.

The RMSProp algorithm has the advantages of fast convergence speed and small oscillation amplitude [14], and its parameter update process is expressed as shown in equation (9), where *θ* is a very small constant.

(9) $$\begin{array}{c} \left\{\begin{array}{c} E_{\text{d}\omega }=\beta E_{\text{d}\omega }+\left(1-\beta \right){\left(\text{d}\omega \right)}^{,2}\\ E_{\text{d}e}=\beta E_{\text{d}e}+\left(1-\beta \right){\left(\text{d}e\right)}^{2},\\ \omega_{i+1}=\omega_{i}-\alpha \frac{\text{d}\omega }{\sqrt{E_{\text{d}\omega }}+\theta },\\ e_{i+1}=e_{i}-\alpha \frac{\text{d}e}{\sqrt{E_{\text{d}e}}+\theta }. \end{array}\right. \end{array}$$

Adaptive moment estimation (Adam) optimization algorithm combines the momentum gradient descent algorithm and the RMSProp algorithm, which can reduce the oscillation amplitude and accelerate the convergence speed of the network [15]. The Adam optimization algorithm was used to update the parameters. The parameter update process during the initial training of the Adam optimization algorithm is expressed as follows:

(10) $$\begin{array}{c} \left\{\begin{array}{c} D_{\text{d}\omega }=\beta_{1}D_{\text{d}\omega }+\left(1-\beta_{1}\right)\text{d}\omega ,\\ D_{\text{d}e}=\beta_{1}D_{\text{d}e}+\left(1-\beta_{1}\right)\text{d}e,\\ E_{\text{d}\omega }=\beta_{2}E_{\text{d}\omega }+\left(1-\beta_{2}\right){\left(\text{d}\omega \right)}^{2},\\ E_{\text{d}e}=\beta_{2}E_{\text{d}e}+\left(1-\beta_{2}\right){\left(\text{d}e\right)}^{2}. \end{array}\right. \end{array}$$

At the *t*-th iteration, the cumulative amount of the modified gradient is expressed as follows:

(11) $$\begin{array}{c} \left\{\begin{array}{c} D_{\text{d}\omega }^{n}=\frac{D_{\text{d}\omega }}{\left(1-\beta_{1}{}^{t}\right)},\\ D_{\text{d}e}^{n}=\frac{D_{\text{d}e}}{\left(1-\beta_{1}{}^{t}\right)},\\ E_{\text{d}\omega }^{n}=\frac{E_{\text{d}\omega }}{\left(1-\beta_{2}{}^{t}\right)},\\ E_{\text{d}e}^{n}=\frac{E_{\text{d}e}}{\left(1-\beta_{2}{}^{t}\right)}. \end{array}\right. \end{array}$$

The parameters are updated according to the momentum and RMSProp algorithm, which are expressed as follows:

(12) $$\begin{array}{c} \left\{\begin{array}{c} \omega_{i+1}=\omega_{i}-\alpha \frac{D_{\text{d}\omega }^{n}}{\sqrt{E_{\text{d}\omega }^{n}}+\theta }.\\ e_{i+1}=e_{i}-\alpha \frac{D_{\text{d}e}^{n}}{\sqrt{E_{\text{d}e}^{n}}+\theta }. \end{array}\right. \end{array}$$

In equations (9)-(12), *β*_1_ and *β*_2_ are 0.9 and 0.999, respectively, *θ* is 10^−8^, *y*_*i*_ is the corresponding target output, and *h*_0_(*x*_*i*_) is the corresponding model probability output of *x*_*i*_.

### 2.3. Analysis of Reconstruction Performance of MRI Image Super-Resolution Algorithm Based on Deep CNN Algorithm

To avoid the impact of loss function, SRCNN still uses the same loss function as DCNN. The quality of the reconstructed image is evaluated regarding peak signal-to-noise ratio (PSNR) and structural similar image metric (SSIM). PSNR is commonly used to evaluate the differences between the image to be estimated and the ideal image, and its calculation equation is as follows:

(13) $$\begin{array}{c} \text{PSNR}\left(f,g\right)=10\;\log_{10}\left(\frac{L^{2}}{\text{MSE}\left(f,g\right)}\right), \end{array}$$

where *L* is the peak signal, *f* is the ideal image, *g* is the image to be estimated, MSE(*f*, *g*) is the mean square error of the image, MSE(*f*, *g*)=1/MN∑_*i*=1_^*M*^∑_*j*=1_^*N*^(*f*(*i*, *j*) − *g*(*i*, *j*))^2^, and *M *×* N* is the size of the image to be estimated.

The structural similarity (SSIM) evaluation result is similar to the human senses, which is calculated as follows:

(14) $$\begin{array}{c} \text{SSIM}\left(f,g\right)={\left(L\left(f,g\right)\right)}^{\alpha }\cdot {\left(C\left(f,g\right)\right)}^{\beta }•{\left(S\left(f,g\right)\right)}^{\gamma }, \end{array}$$

where *μ*_*f*_, *μ*_*g*_, *σ*_*f*_, and *σ*_*g*_ are the mean values and standard deviations of the ideal image *f* and the image *g* to be evaluated, respectively, *σ*_*fg*_ is the covariance of *f* and *g*, *c*_1_=(*k*_1_  *R*)^2^, *c*_2_=(*k*_2_*R*)^2^, *R* is the range of image pixel values, *k*_1_ and *k*_2_ are 0.01 and 0.03, respectively, *c*_3_=*c*_2_/2, *α*=*β*=*γ*=1, and *L*(*f*, *g*), *C*(*f*, *g*), and *S*(*f*, *g*) represent image brightness, structure, and contrast, respectively.

### 2.4. Knee MRI Examination and Diagnostic Criteria

1.5 T superconducting MRI (Siemens, Germany) was used to examine the patient that was in the supine position, the knee joint was naturally externally rotated 25° during the examination, and the knee joint was fixed during the scan. The scanning layer thickness was 3 mm, the layer spacing was 0.2∼0.4 mm, the matrix was 256×256, and the joint space was used as the scanning center. All patients underwent coronal and sagittal scans. The repetition time (TR) of T2WI was 800–1000 ms, and the echo time (TE) was 26 ms. The spin echo sequence T1WI had TR of 450–500 ms and TE of 14 ms. MRI diagnostic criteria were as follows: all patients' MRI scan images were individually read by three radiologists with senior titles, who provided reports to evaluate the lateral meniscus injury and its damage morphology.

### 2.5. Surgical Methods and Observation Indicators

Schatzker classification standard in the study of Kumar et al. [16] was referred, and the types of platform fractures of MRI images of all patients in the study were classified into six types. Different types of platform fractures received different surgical treatments.

The grading standard of meniscus injury was as follows. Grade 1: there is a patchy signal, showing mild degeneration. Grade 2: there is a linear signal, showing serious degeneration. Grade 3: there is a linear signal, showing a meniscus tear [17]. All patients were scored according to Lysholm knee joint function score before and after surgery, and the changes of knee joint function scores before and after treatment were compared to analyze the effect of surgical treatment.

### 2.6. Statistical Methods

The test data were processed using SPSS 19.0. The results of intraoperative exploration or arthroscopy were used as the standard to analyze the accuracy of MRI diagnosis. Enumeration data were expressed as a percentage (%), tested by the *χ*^2^ test. *P* < 0.05 indicated that the difference was statistically considerable.

## 3. Results

### 3.1. The Influence of Loss Function and Number of Convolution Kernels on Reconstruction Performance

The comparison of training curves of the three loss functions is shown in Figure 2. PSNRs of the three loss functions all increased first and then became stable with the increase of the number of iterations. The PSNR of the mean square error loss function was relatively higher under the same number of iterations, and the convergence was relatively faster during the training.

PSNRs of MRI reconstructed images under different numbers of convolution kernels are compared in Figure 3. With the increase of the number of iterations, the PSNR of the MRI reconstructed image under different convolutions and numbers showed a state of increasing first and then being stable in a certain region. As the number of convolution kernels increased, the PSNR of the MRI reconstructed image increased significantly. The number of convolution kernels was increased from 1 to 3, and the PSNR of the MRI reconstructed image was increased by 0.68 dB. The number of convolution kernels was increased from 3 to 5, and the PSNR of the MRI reconstructed image was increased by 0.16 dB.

### 3.2. Quality Analysis of Reconstructed MRI Image

PSNR value of the SRCNN algorithm was compared with the average PSNR value of DCNN, cubic spline interpolation, and deeply recursive convolutional network (DRCN) based on the residual learning algorithm (Figure 4). The PSNR of the SRCNN algorithm was (42.19 ± 4.37) dB, which was greatly higher than that of other algorithms, and the difference was remarkable (*P* < 0.05).

The average SSIMs of different algorithms were compared (Figure 5). The average SSIM of DCNN, cubic spline interpolation, DRCN, and SRCNN algorithms was 0.9447, 0.9316, 0.9764, and 0.9951, respectively. The SSIM of SRCNN algorithm was notably higher than that of other algorithms, and the difference was substantial (*P* < 0.05).

### 3.3. MRI Diagnosis Results of Meniscus Injury

The MRI results of patients with meniscus injury before and after treatment were analyzed (Figure 6). The normal meniscus MRI image showed uniform low signal and regular shape (Figure 6(a)). The MRI signal of meniscus injury patients showed focal ellipse or round high signal, which did not touch the articular surface of the meniscus (Figure 6(b)). The horizontal linear hyperintensity shadow extended to the edge of the joint capsule of the meniscus but did not exceed the articular surface of the meniscus (Figure 6(c)). In addition, there was an irregular high signal shadow in the meniscus (Figure 6(d)).

### 3.4. MRI Diagnosis Result of Meniscus Injury Degree

The results of arthroscopy or intraoperative exploration were used as the gold standard to evaluate the accuracy of MRI in the diagnosis of meniscus injury (Figure 7). There were 19 cases (31.67%), 34 cases (56.67%), and 7 cases (11.67%) of meniscus injury diagnosed by arthroscopy as grades I, II, and III, respectively. There were 20 cases (33.33%), 27 cases (45.99%), and 13 cases (21.67%) of meniscus injuries diagnosed by MRI as grades I, II, and III, respectively. There was no obvious difference in the grading of meniscus injury between results of MRI and arthroscopy (*P* > 0.05).

### 3.5. Statistics of Treatment Methods of MRI-Diagnosed Meniscus Injury

According to the degree and type of meniscus injury, different treatment methods were implemented for the 60 patients included in the study, and the proportion of patients in different methods was calculated (Figure 8). Seventeen cases (28.33%) were treated with meniscus suture, 39 cases (65.00%) underwent secondary resection, 3 cases (5.00%) underwent partial resection, and 1 case (1.67%) underwent total resection.

### 3.6. Knee Function Scores of Patients Treated with Different Methods before and after Treatment

The knee function scores of patients with different treatment methods were compared before and after treatment (Figure 9). There was no statistical difference in the knee function scores of all patients before treatment (*P* > 0.05). After meniscus suture, secondary resection, partial resection, and total resection were used to treat meniscus injury patients, and the knee function scores were (83.17 ± 8.63), (80.06 ± 7.96), (84.34 ± 7.74), and (85.52 ± 5.97), respectively. In addition, there was no great difference in the knee function scores among patients treated by different treatment methods after treatment (*P* > 0.05). The knee function scores of each group after treatment were significantly different from those before treatment (*P* < 0.01).

## 4. Discussion

The entire training process of SRCNN based on the deep CNN algorithm was calculating this round of loss according to the loss function after all levels and processing are passed through the input previous to the propagation. In this research, appropriate optimization methods such as stochastic gradient descent was adopted to update the parameters of each layer in the direction of reducing the loss. Therefore, the loss function was the instructor of the entire network learning, which had a great influence on the quality of the final learning result [18]. Then, the training curves of the three commonly used loss functions were compared. It was found that the PSNR of the mean square error loss function was high, and the convergence was fast during the training. The mean square error loss function belongs to the pixel-by-pixel loss function, which can well converge to the local minimum [19]. Therefore, the mean square error loss function was selected as the loss function. The depth of CNN has a great impact on network performance, and the depth of SRCNN is mainly determined by the number of convolution kernels in the network [20]. PSNRs of MRI reconstructed images under different numbers of convolution kernels were compared. It was found that as the number of convolution kernels increased, the PSNR of the MRI reconstructed image increased significantly. The number of convolution kernels was increased from 1 to 3, and the PSNR of the MRI reconstructed image was increased by 0.68 dB. The number of convolution kernels was increased from 3 to 5, and the PSNR of the MRI reconstructed image was increased by 0.16 dB. These results indicated that the PSNR increased with the increase in the number of S3D-RDBs, suggesting that the quality of the MRI images reconstructed by the SRCNN network was getting better and better. It was because the more the number of convolution kernels in the SRCNN network, the deeper the network depth, which can capture more feature maps of different levels to highlight more detailed information [21]. As the number of convolution kernels increased, the increase in PSNR became small. It may be because as the network deepened, information loss still occurred when information was transmitted in the network, which made the backpropagation of the gradient in the network more difficult [22].

Meniscus injury has a significant correlation with the stability of the knee joint, postoperative inflammation, and other complications [23]. Iqbal et al. [24] found that MRI diagnosis of articular surface collapse was consistent with the arthroscopic diagnosis. In this research, the results showed that the different degrees of MRI meniscus injury were not statistically significant with the results of arthroscopy (*P* > 0.05). It showed that there were still a small number of false positives and false negatives in MRI diagnosis. It may be related to the uneven confounding signal of connective tissues such as synovium and muscle health, which led to artifacts of meniscus damage during MRI scan. However, there was no considerable difference between MRI diagnosis results and arthroscopic diagnosis results, indicating that MRI had a certain potential value in the diagnosis of meniscus injury. Lu et al. [25] pointed out that arthroscopy had the characteristics of less surgical trauma and fast recovery speed and is used in the clinical treatment of meniscus injuries. Based on the imaging characteristics, different methods were used to treat patients with different degrees of meniscus injury. The results showed that there was no great difference in knee function scores among patients treated by different treatment methods after treatment (*P* > 0.05). The knee function scores of each group after treatment were significantly different from those before treatment (*P* < 0.01), which suggested that the effect of arthroscopic surgery on knee meniscus injury was significant.

## 5. Conclusion

Based on the deep CNN algorithm, the Adam optimization algorithm was introduced to optimize it, which was then applied to the knee joint meniscus injury diagnosis. The clinical effect of arthroscopic surgery in knee meniscus injury based on MRI images was evaluated. The results revealed that SRCNN based on deep CNN algorithm significantly improved the quality of knee MRI images. However, there are still some shortcomings in this research, which does not perform a statistical analysis on the parameters and calculation cost of the algorithm in MRI image processing. In the future work, we will further analyze it to clarify the value and significance of SRCNN based on deep CNN algorithm in the diagnosis of knee meniscus injury. In summary, the SRCNN algorithm based on the deep convolutional network algorithm improved the MRI image quality and the diagnosis of knee meniscus injuries. Moreover, arthroscopic knee surgery had good results and had great clinical application and promotion value.

## Figures and Tables

**Figure 1:** SRCNN processing flow for low-resolution image.

**Figure 2:** Comparison of training curves with the same loss function.

**Figure 3:** The influence of the number of convolution kernels on reconstruction performance.

**Figure 4:** Comparison of PSNR of reconstructed MRI images with different algorithms.

**Figure 5:** Comparison of SSIM of reconstructed MRI images with different algorithms.

**Figure 6:** MRI image of meniscus. (a) MRI image of normal meniscus. (b) MRI image of grade I injury in the posterior horn of the medial meniscus (female, 24 years old). (c) MRI image of grade II injury of the posterior horn of the medial meniscus (female, 62 years old). (d) MRI image of grade III injury of the posterior horn of medial meniscus (male, 36 years old).

**Figure 7:** Analysis of the accuracy of MRI in the diagnosis of meniscus injury.

**Figure 8:** Statistics of treatment methods of MRI-diagnosed meniscus injury.

**Figure 9:** Comparison of knee joint function scores of patients with different treatment methods before and after treatment (^*∗*^^*∗*^indicated a significant difference versus that before treatment, *P* < 0.01).

## Data Availability

The data used to support the findings of this study are available from the corresponding author upon request.
